# Nanocurcumin Improves Lipid Status, Oxidative Stress, and Function of the Liver in Aluminium Phosphide-Induced Toxicity: Cellular and Molecular Mechanisms

**DOI:** 10.1155/2022/7659765

**Published:** 2022-09-12

**Authors:** Ali Salimi, Nejat Kheiripour, Ali Fathi Jouzdani, Hassan Ghasemi, Sara Soleimani Asl, Abolfazl Ghafouri-Khosrowshahi, Akram Ranjbar

**Affiliations:** ^1^Medicinal Plants and Natural Products Research Center, Hamadan University of Medical Sciences, Hamadan, Iran; ^2^Research Center for Biochemistry and Nutrition in Metabolic Diseases, Kashan University of Medical Sciences, Kashan, Iran; ^3^Student Research Committee, Hamadan University of Medical Science, Hamadan, Iran; ^4^USERN Office, Hamadan University of Medical Science, Hamadan, Iran; ^5^Department of Clinical Biochemistry, Abadan School of Medical Sciences, Abadan, Iran; ^6^Department of Anatomical Sciences, Faculty of Medicine, Hamadan University of Medical Sciences, Hamadan, Iran; ^7^Departments of Medicinal Chemistry and Pharmacology and Toxicology, School of Pharmacy, Hamadan University of Medical Sciences, Hamadan, Iran; ^8^Nutrition Health Research Center, Hamadan University of Medical Sciences, Hamadan, Iran

## Abstract

**Background:**

The present study aimed to evaluate the effect of nanocurcumin and curcumin on liver transaminases, lipid profile, oxidant and antioxidant system, and pathophysiological changes in aluminium phosphide (ALP) induced hepatoxicity. *Material and Methods*. In this experimental study, thirty-six male Wistar rats were randomly divided into six groups curcumin (Cur), nanocurcumin (Nanocur), ALP, ALP+Cur, and ALP+Nanocur. All treatments were performed by oral gavage for seven days. After treatment, animals were sacrificed, and liver and blood samples were taken. Serum levels of aspartate aminotransferase (AST), alanine transaminase (ALT), alkaline phosphatase (AP), total bilirubin, cholesterol, triglyceride, high-density lipoprotein (HDL), low-density lipoprotein (LDL), and very-low-density lipoprotein (VLDL) were measured by photometric methods. Total antioxidant capacity (TAC) and malondialdehyde (MDA) as parameters of oxidative stress and mRNA expression of the nonenzyme protein including Sirtuin 1 (STR1), Forkhead box protein O1 (FOXO1) and protein O3 (FOXO3), catalase (CAT), and glutathione peroxidase (GPX) as the enzyme protein in homogenized tissues have been investigated. A histologist analyzed liver tissue sections after staining with hematoxylin-eosin.

**Results:**

In the aluminium phosphide group, there was a significant increase in MDA, ALT, AST, and AP and total bilirubin, cholesterol, triglyceride, LDL, and VLDL; AST, ALT, total bilirubin, LDL, VLDL, cholesterol, and MDA were significantly decreased; and HDL and TAC were significantly increased compared to ALP (*P* < 0.05). In the ALP+Nanocur group, ALT, AST, ALP, total bilirubin, cholesterol, LDL, VLDL, triglyceride, and MDA were significantly decreased and HDL and TAC were increased significantly (*P* < 0.05). The effect of nanocurcumin on controlling serum levels of LDL, VLDL, triglyceride, and MDA in ALP-poisoned rats was significantly more than curcumin (*P* < 0.05). The ALP group had significant changes in genes *SIRT1*, *FOXO1a*, *FOXO3a*, *CAT*, and *GPX* compared to healthy controls (*P* < 0.05). Nanocurcumin mice expressed more *SIRT1*, *FOXO1a*, *CAT*, and *GPX* genes than controls, and curcumin-treated mice expressed more *SIRT1* and *FOXO1a* genes (*P* < 0.05). Histopathological findings also indicated a more significant protective effect of nanocurcumin relative to curcumin against ALP-induced hepatotoxicity.

**Conclusion:**

Nanocurcumin significantly protects the liver against aluminum phosphide toxicity. It is suggested that nanocurcumin-based drugs be developed to reduce the toxic effects of ALP in poisoned patients.

## 1. Introduction

Aluminium phosphide (ALP) is a potent suicide tool which is widely utilized. Despite high mortality rates and supportive treatment, including the rapid decontamination and resuscitative measures, the exact mechanisms of acute toxicity are not fully understood. Rice tablet or ALP is one of the metal phosphides widely used in some countries [1]. ALP is a dark grey chemical compound that is also available in the form of yellow crystals. It is used for industrial and agricultural purposes to preserve rice and other stored grains or animals' feeds [2]. This compound is available under different trade names such as Phostoxin, Celphos, Quickphos, Phostek, and Bhostoxin [3]. ALP leads to many intentional/accidental poisoning and deaths [4]. About 300,000 deaths from pesticide poisoning are reported worldwide annually [5]. Unfortunately, even consuming tiny amounts of this toxin can lead to death [6]. When exposed to water and moisture, ALP produces phosphine (PH3)—a colourless, flammable, toxic gas—ammonia, and carbon dioxide. After oral consumption, it reacts with gastric acid and creates phosphine gas readily absorbed through the gastrointestinal tract and the lung epithelium [7]. The precise mechanism of phosphine gas toxicity in humans has not been fully understood. Multiorgan failure is finally caused by the severe cellular damage brought on by ALP [8]. In the mitochondria, phosphorus gas blocks cytochrome oxidase C. [9]. Inhibition of this respiratory chain component results in oxidative-stress in the cell and an increase in the generation of free radicals [9]. Phosphine gas also inhibits cellular peroxidase, leading to increased production of free radicals [10]. The target organs for phosphine intoxication include the lung, heart, brain, digestive tract, kidney, and liver. The liver is one of the essential target organs in ALP poisoning. It was shown that most deaths occurring after the first 24 hours of ALP poisoning are in terms of the hepatotoxicity [11, 12]. Aspartate aminotransferase (AST), alanine aminotransferase (ALT), and alkaline phosphatase are enzymatic markers of liver damage [13]. On the other hand, the liver plays an important role in detoxification and lipid and lipoprotein metabolism. Hence, in the case of liver toxicity and damage, the level of these factors may dysregulate [14]. High-density lipoproteins (HDL), low-density lipoprotein (LDL), and very-low-density lipoprotein (VLDL) are the most critical lipoproteins [15]. VLDL is converted to LDL in the lipid transport process by losing triglycerides. HDL transfers cellular cholesterol from other cells to the liver [15]. These molecules may therefore be used as indicators of liver health. Alternatively, oxidative stress plays an important function in hepatotoxicity [16]. SIRT1 downregulation promotes oxidative stress and inflammation in hepatotoxicity. Pieces of evidence indicated that maintenance of SIRT1 in the proinflammatory context and oxidative stress during hepatotoxicity might be clinically relevant [17]. The catalytic activity of SIRT1 is essential in the hepatoprotective effects of polyphenols where SIRT1 inhibitors block and the allosteric SIRT1 activators mimic the hepatoprotective effects of polyphenols [18]. FOXOs are transcription factors which are members of the Forkhead family, among which FOXO1 and FOXO3 are the most common. When FOXOs move into the nucleus and activate their protein expression, they start various cellular functions, including inhibiting oxidative stress [19]. The SIRT1 and FOXO connection are implicated in resistance to oxidative stress [20]. The reactive oxygen species (ROS) can be neutralized in organisms by a tiny thiol molecule called glutathione (GSH) and enzymes including catalase (CAT) and glutathione peroxidase (GPx) as well as antioxidant dietary components [21]. There is no specific antidote to treat ALP poisoning, only supportive treatment is provided [22]. However, studies showed that administration of antioxidant compounds and other supportive therapies such as oxygen, electrolytes, etc., can be beneficial to prevent oxidative damage caused by free radicals and peroxidation in tissues, especially in the liver. Studies have shown that vitamin E administration may effectively prevent phosphine-induced liver injury by inhibiting lipid peroxidation [7]. There is increasing evidence that plant complexes and their isolated components may influence oxidative stress and liver toxicity, and may serve as antidotes for certain situations, such as ALP-induced toxicity [23–26]. Therefore, focusing on traditional medicine and herbal remedies to achieve natural, inexpensive antioxidant drugs with minimal side effects and superior impact is needed [27]. Some herbs are considered a rich source of natural antioxidants [28]. Curcumin is a polyphenolic compound and an active pigment in the roots of *Curcuma longa* L. (Turmeric) [29]. Curcumin has healing properties for various diseases, such as cancer, pulmonary disease, neurodegenerative diseases, kidney disease, metabolic disorders, heart disease, and inflammatory diseases. Curcumin has anti-inflammatory, antioxidant, wound healing and antimicrobial activity [30]. However, curcumin's limitations are insolubility, low tissue distribution and uptake, low action, rapid metabolism, and inactivation of products in the body [31]. Curcumin is highly sensitive to physiological pH changes in the body. Besides, it is poorly absorbed by the acidic environments of the digestive tract [32]. Various solutions were proposed to overcome these limitations. These include adjuvants such as piperine, design of structural analogues such as EF-24, metabolism inhibitors, phospholipid complex curcumin, liposomal curcumin, and curcumin nanoparticles [33]. It can be suggested that curcumin-Au@ZnO nanoparticles could inhibit *Staphylococcus aureus* from producing *α*-hemolysin toxin. It seems that in the future, these nanoparticles can be used in biomedical and pharmaceutical applications [34]. Furthermore, endosomal nanocurcumin is a polydisperse colloidal suspension in which hydrophobic nanocurcumin particles are incorporated into micelles resulting in increased water solubility and bioavailability (29 centrosomes are oleic acid-derived branched polymeric nanocarriers). These carriers' characteristics include stability, nontoxicity, neutrality, biodegradability, easy preparation, and low cost of production [31, 35]. It can be suggested that curcumin can be a viable treatment option to detoxify ALP-induced toxicity, particularly hepatotoxicity. As curcumin becomes nanoscale and its antioxidant properties increase, its effectiveness may also be enhanced. The present study is aimed at evaluating the effect of nanocurcumin and curcumin on liver transaminases, lipid profile, oxidant and antioxidant system, mRNA expression, and pathophysiological changes in ALP-induced hepatoxicity.

## 2. Materials and Methods

### 2.1. Chemicals and Reagents

Curcumin and endosomal nanocurcumin were ordered from Exir Nano Sina Co. (Iran). ALP (photo in, 3 mg tablet, ALP 56%, w/w) was purchased from Shanghai, AgroChina International Company (Ltd., China). All other used chemicals and reagents were fresh and highest commercial grade prepared from Sigma® (USA).

### 2.2. Animals and Experimental Design

Thirty-six adult male Wistar rats weighing 220–250 g were selected from the animal house of Hamadan University of Medical Sciences. Animals were maintained in standard cages (3 animals per cage) with wood shavings bedding under optimum conditions of temperature (22-27° C), humidity (60 5 5%), and light (12 h light and 12 cycles). Animals were given ad libitum access to food and water. All procedures were conducted by the ethical principles of working with laboratory animals at Hamadan University of Medical Sciences. The animals were allowed to adapt to the environment one week before the experiments began. Animals were then randomly divided into six groups (*n* = 6) and treated as follows: the first group, the control group, received no treatment; the second group, the curcumin (Cur) group, received 100 mg/kg/day of curcumin; the third group, the nanocurcumin (Nanocur) group, received 100 mg/kg/day; the fourth group, the ALP group, received 2 mg/kg/day of ALP; the fifth group, the ALP+Cur group, received 100 mg/kg/day of curcumin plus 2 mg/kg/day of ALP; and the sixth group, the ALP+Nanocur group, received 100 mg/kg/day of nanocurcumin plus 2 mg/kg/day of ALP. All treatments were performed by oral gavage for seven consecutive days. Our previous study served as the basis for selecting doses.

### 2.3. Sampling

Twenty-four hours after the last treatment, animals were euthanized with ketamine (50 mg/kg) under deep anaesthesia. Blood samples (3–5 ml) were taken directly from the heart (5 ml syringes). Serum of blood samples was isolated by centrifuge method (15 min at 5000 rpm) and stored at -20° C for lipid profile and liver injury markers measurement. The liver tissues were isolated and washed with normal saline. Tissue specimens were divided into two parts, one part was frozen in liquid nitrogen and maintained at −80°C until biochemical measurements, and the other part was maintained in 10% formalin at 2–8°C for histopathological examinations. For measuring biochemical parameters, liver tissues were homogenized in a lysis buffer consisting of 10 mM HEPES, 10 mM KCl, 1.5 mM MgCl2, 1.0 mM EDTA, Triton X-100 0.2%, and 0.5 mM DTT. Afterwards, the resulting solution was centrifuged at 14,000 rpm at 4°C; the supernatant was removed and used for biochemical measurements or stored at −20°C for future use.

### 2.4. Measurement of Total Protein

Total protein was measured by the Bradford method using Coomassie Brilliant Blue G-250. Briefly, 100 mg Coomassie Blue was dissolved in 100 ml methanol (50% v/v) and 100 ml phosphoric acid (85% w/v). After completely dissolving, the resulting solution was diluted to 1 L with deionised water and filtered through Whatman filter paper No.1. The protein content of samples was determined by adding 10 ml of homogenized tissues to 190 *μ*l of reagent. The absorbance of samples and standards was read in 590 nanometers [36].

### 2.5. Measurement of Malondialdehyde (MDA)

The photometric method measured the levels of malondialdehyde as a marker of lipid peroxidation. Briefly, 100 *μ*l H2SO4 (0.05 M), 1.5 ml trichloroacetic acid 20%, 1.5 ml thiobarbituric acid, and 200 *μ*l of water were added to 100 *μ*l of homogenized tissue supernatant. The reaction mixture was placed at 95°C for 60 min. Then, 3 ml of n-butanol was added to the reaction mixture and was shaken vigorously. After centrifugation (1,000 g, 10 min), the butanol layer was removed. The absorbance of samples and standard (tetra ethoxy propane) was read in 532 nanometers. MDA levels were expressed as nmol/mg protein [37].

### 2.6. Measurement of Total Antioxidant Capacity (TAC)

The FRAP (Ferric Reducing Ability of Plasma) method measured total antioxidant capacity. Briefly, 100 *μ*l of homogenized tissue supernatant tissue was added to 3 ml of FRAP reagent. FRAP reagent made using 25 ml acetate buffer (300 mM, pH =3.6), 16 ml acetic acid per buffer unit, 2.5 ml TPTZ solution (TPTZ 10 mM in HCl 40 mM), and 2.5 ml FeCl_3_.6H_2_O. Subsequently, the resulting solution was vortexed and incubated at 37°C for 10 min, and its absorption was read at a wavelength of 593 nm. TAC levels were expressed as nmol/mg protein [38].

### 2.7. AST Measurement

Serum AST levels were measured by the photometric method. Reagents 1 and 2 were mixed (4 : 1 ratio) to produce the final reagent. Reagent 1 included TRIS (pH =7.8, 80 mmol/l), L-aspartate (240 mmol/l), malate dehydrogenase (≥600 U/l) and lactate dehydrogenase (≥600 U/l). Reagent 2 consisted of 2-oxoglutarate (2 mmol/l) and NADH (0.18 mmol/l). Next, 20 *μ*l of the serum sample was transferred into a clean cuvette containing 1000 *μ*l of final reagent. Optical absorption of the reaction mixture was measured at a wavelength of 340 nm immediately and in 1, 2 and 3 min after preparation of the reaction mixture. Finally, serum AST levels were measured in U/l using the following formula: *Δ*A/min ∗ 1890 = AST (U/L).

### 2.8. ALT Measurement

Serum ALT levels were measured by the photometric method. Reagents 1 and 2 were mixed (4 : 1 ratio) to produce the final reagent. Reagent 1 included TRIS (pH =7.5, 100 mmol/l), L-Alanine (500 mmol/l), and lactate dehydrogenase (≥1200 U/l). Reagent 2 consisted of 2-oxoglutarate (15 mmol/l) and NADH (0.18 mmol/l). Next, 20 *μ*l of the serum sample was transferred into a clean cuvette containing 1000 *μ*l of the final reagent. Optical absorption of the reaction mixture was measured at the wavelength of 340 nm immediately and in 1, 2 and, 3 min after preparation of the reaction mixture. Finally, serum ALT levels were measured using the following formula: ΔA/min∗1750 = ALT (U/L).

### 2.9. Alkaline Phosphatase Measurement

Serum alkaline phosphatase level was measured using the photometric method. The final reagent was made by mixing reagents 1 and 2. Reagent 1 consisted of diethanolamine (pH =9.8, 1 mol/l) and magnesium chloride (0.5 mmol/l). Reagent 2 contained P-nitrophenyl phosphate (10 mmol/l). Afterwards, 20 *μ*l of the serum sample was transferred into a clean cuvette containing 1000 *μ*l of the final reagent. Optical absorption of the reaction mixture was measured at the wavelength of 405 nm immediately and in 1, 2, and 3 min after preparation of the reaction mixture. The difference in reading absorbance was measured at 1, 2, and 3 min compared to the preceding time. The mean of absorption differences was multiplied by the 2757 factor. Finally, serum alkaline phosphatase was expressed in U/l.

### 2.10. Total Bilirubin Measurement

Serum total bilirubin level was measured using reagents 1 and 2 and a calibrator. Reagent 1 consisted of Phosphate Buffer (40 mmol/l), sodium chloride (9 g/l), detergent and a stabilizer. Reagent 2 consisted of 2,4-chlorophenyl-diazonium salt (1 mmol/l), hydrochloric acid (30 mmol/l) and detergent. In the first step, 25 *μ*l of serum or calibrator was transferred into a clean cuvette, and 1000 *μ*l of the reagent one was added. After mixing for 5 minutes and incubation at 37°C for 5 min, the direct optical absorption of the sample and calibrator was measured at 546 nm. Afterwards, 250 *μ*l of reagent two was added to the mixture. After mixing for 5 minutes and incubation at 37°C for 5 min, the secondary optical absorption of the sample and calibrator were measured. Finally, total bilirubin was measured according to the following formula: Bili.T (mg/dl) = Δ*A* Sample/Δ*A* Calibrator∗Concentration of Calibrator (*mg*/*dl*).

### 2.11. Triglyceride Measurement

Serum triglyceride levels were measured by the photometric method using a reagent and calibrator. Reagent consisted of goods buffer (pH =7.2, 50 mmol/l), 4-chlorophenol (4 mmol/l), ATP (2 mmol/l), Mg^2+^ (15 mmol/l), glycerol kinase (≥0.4 KU/l), peroxidase (≥2 KU/l), lipoprotein lipase (≥2 KU/l), 4-amino antipyrine (0.5 mmol/l), and glycerol-3-phosphate-oxidase ((≥0.5 KU/l). In the first step, 10 *μ*l of the serum or calibrator was added to 1000 *μ*l of the reagent in a clean cuvette. After mixing for 5 minutes and incubation at 37°C for 5 min, the optical absorption of the sample and calibrator was measured at 505 nm. Serum triglyceride levels were measured using the following formula: TG (mg/dl) = *A* *Sample*/*A* Calibrator∗Concentration of Calibrator (mg/dl).

### 2.12. Total Cholesterol Measurement

Serum total cholesterol levels were measured using a reagent and calibrator. The reagent included goods buffer (pH =6.7, 50 mmol/l), phenol (5 mmol/l), 4-amino antipyrine (0.3 mmol/l), cholesterol esterase (≥200 lU/l), cholesterol oxidase (50 U/l), and peroxidase (3 KU/l).

First, 10 *μ*l of the serum or calibrator was added to 1000 *μ*l of the reagent in a clean cuvette. After mixing and incubation at 37°C for 10 min, the optical absorption of the sample and calibrator was measured at 546 nm. Serum total cholesterol levels were measured using the following formula: T.Chol (mg/dl) = *A* Sample/*A* Calibrator∗Concentration of Calibrator (mg/dl).

### 2.13. HDL Measurement

Serum HDL levels were measured using reagents 1 and 2 and a calibrator. Reagent 1 included goods buffer (pH =7.0, 26 mmol/l), 4-amino antipyrine (0.6 mmol/l), peroxidase (1600 U/l), ascorbate oxidase (1800 U/l), and antihuman *β*–lipoprotein antibody (sheep). Reagent 2 consisted of goods buffer (pH =7.0, 26 mmol/l), cholesterol esterase (800 U/l), cholesterol oxidase (4000 U/l), N-ethyl-N-(2-hydroxy-3-sulfopropyl)-3,5-dimethoxy-4-fluoroaniline (0.16 mmol/l), and sodium salt. First, 10 *μ*l of serum or calibrator was transferred into a clean cuvette, and 1000 *μ*l of the reagent one was added. After mixing and incubation at 37°C for 5 min, the direct optical absorption of the sample and calibrator was measured at 600 nm. Afterwards, 250 *μ*l of reagent 2 was added to the mixture. After mixing and incubation at 37°C for 5 min, the secondary optical absorption of the sample and calibrator were measured. Finally, HDL was measured according to the following formula: HDL (mg/dl) = *A* Sample/*A* Calibrator∗Concentration of Calibrator (mg/dl).

### 2.14. LDL and VLDL Measurement

Serum total bilirubin levels were measured using reagents 1 and 2 and a calibrator. Reagent 1 contains goods buffer (pH =6.8, 22 mmol/l), cholesterol esterase (≥2 KU/l), cholesterol oxidase (≥2 KU/l), N-(2-hydroxy-3-sulfopropyl)-3,5-dimethylaniline (0.43 mmol/l), and catalase (≥400 KU/l). Reagent 2 consisted of goods buffer (pH =0.7, 22 mmol/l), 4-amino antipyrine (0.68 mmol/l), peroxidase (≥3 KU/l), and sodium azide. First, 10 *μ*l of serum or calibrator was transferred into a clean cuvette, and 1000 *μ*l of reagent 1 was added.

After mixing and incubation at 37°C for 5 min, the direct optical absorption of the sample and calibrator was measured at 650 nm. Afterwards, 250 *μ*l of reagent two was added to the mixture. After mixing and incubation at 37°C for 5 min, the secondary optical absorption of the sample and calibrator were measured. Serum LDL levels were measured using the following formula: LDL (mg/dl) = *A* Sample/*A* Calibrator∗Concentration of Calibrator (mg/dl). Serum VLDL levels were converted using the following formula: VLDL − *C* = TC–(LDL − *C* + HDL − *C*).

### 2.15. Determination of mRNA expression of SIRT1, FOXO1, FOXO3, CAT and GPX in the brain tissue

Total RNA extraction was performed manually from tissues by RNX-Plus reagent (Cinnagen, Tehran, Iran). Complementary DNA (cDNA) synthesis was carried out by the PrimeScript RT reagent kit (TaKaRa Biotechnology, Japan). Quantitative Real-Time PCR was performed with SYBR premix Ex TaqTM II (TaKaRa Biotechnology, Japan) on a Roche Light Cycler 96 System (Roche Life Science Deutschland GmbH, Sandhofer, Germany). The characteristics of the forward and reverse primer sequence (5′ →3′) were listed as follows: *β*-Actin forward: CCCGCGAGTACAACCTTCT, and reverse: CGTCATCCATGGCGAACT; SIRT1 forward: CAGTGTCATGGTTCCTTTGC, and reverse: CACCGAGGAACTACCTGAT; FOXO1a; forward: CGAGTGGATGGTGAAGAGTG, and reverse: CGAATAAACTTGCTGTGTAGGG; FOXO3a forward: CTCCCGTCAGCCAGTCTATG, and reverse: GCTTAGCACCAGTGAAGTTCC; CAT forward: CCCAGAAGCCTAAGAATGCAA, and reverse: TCCCTTGGCAGCTATGTGAGA; GPX forward: CACTGTGGCTGAGCTGTTGT, and reverse: CCAAGCAATTCAAGCCTCT. To investigate the fold change in gene expression, the 2 − ΔΔ*CT* formula was used [39]. At that time, 10 *μ*l of H_2_O diluted sample was added to 300 ml reagent warmed at 37°C. Then, 100 *μ*L of liver tissue sample was added to 3 ml of FRAP reagent. The complex between TPTZ and Fe_2_+ makes a blue colour with 593 nm absorbance.

### 2.16. Histopathological Examination

The liver tissue of rats was fixed in 10% formalin at 2–8°C for a week. Then, tissues were dehydrated in 50%, 70%, 96%, and 100% ethanol concentrations. The tissues were placed in xylene for 45 minutes to clarify. Afterwards, tissues were immersed in molten paraffin and sections of 4 *μ*m thick were obtained using a microtome. Finally, slides were stained with hematoxylin-eosin dye and evaluated by a histologist.

### 2.17. Statistical Analysis

Data were presented as *mean* ± *SD*. Groups were compared using One-Way ANOVA followed by Tukey's post hoc tests. Mann–Whitney test was used for variables with abnormal distribution. Normality of data distribution was assessed using the Kolmogorov–Smirnov test. Data were analyzed using SPSS V.22 and GraphPad Prism V.6. *P* < 0.05 was considered a significant level.

## 3. Results

### 3.1. Aluminium Phosphide Effect on Biochemical Parameters

Administration of ALP significantly increased serum levels of MDA (*P* < 0.01) (Figure 1(a)), AST (*P* < 0.01), ALT (*P* < 0.001), ALP (*P* < 0.01), and total bilirubin (*P* < 0.01) (Figure 2), TG (*P* < 0.01), T. Chol (*P* < 0.01), LDL (*P* < 0.01), and VLDL (*P* < 0.001) (Figure 3).

in comparison to the control group. Also, ALP administration significantly decreased serum levels of TAC (*P* < 0.01) (Figure 1(b)) and HDL (Figure 3) (*P* < 0.001) compared to the control group.

### 3.2. Curcumin/Nanocurcumin Effect on Biochemical Parameters

The administration of curcumin/nano curcumin alone had no significant effect on any of the biochemical parameters (*P* > 0.05) (Figures 1–3).

### 3.3. Curcumin/Nanocurcumin Effect on MDA in Aluminum Phosphide Toxicity

Liver MDA levels were significantly reduced in the ALP+Cur and ALP+Nanocur groups compared to the aluminum phosphide group (*P* < 0.01). Tissue MDA levels were significantly higher in the ALP+Cur group than in the ALP+Nanocur and control groups (*P* < 0.01), but there was no significant difference between the control and ALP+Nanocur groups in terms of liver MDA (*P* > 0.05) (Figure 1(a)).

### 3.4. Curcumin/Nanocurcumin Effect on TAC in Aluminum Phosphide Toxicity

Liver TAC levels were significantly increased in the ALP+Cur and ALP+Nanocur groups compared to the aluminum phosphide group (*P* < 0.01). There was no significant difference among ALP+Cur, ALP+Nanocur and control groups in terms of liver TAC (*P* > 0.05) (Figure 1(b)).

### 3.5. Curcumin/Nanocurcumin Effect on AST in Aluminum Phosphide Toxicity

Serum AST levels significantly declined in ALP+Cur and ALP+Nanocur groups compared to the aluminum phosphide group (*P* < 0.05). There was no significant difference among ALP+Cur, ALP+Nanocur and control groups in terms of serum AST (*P* > 0.05) (Figure 2(a)).

### 3.6. Curcumin/Nanocurcumin Effect on ALT in Aluminum Phosphide Toxicity

Serum ALT levels were significantly decreased in ALP+Cur (*P* < 0.05) and ALP+Nanocur (*P* < 0.01) groups compared to the ALP group (*P* < 0.05). There was no significant difference among ALP+Cur, ALP+Nanocur and control groups in terms of serum ALT (*P* > 0.05) (Figure 2(b)).

### 3.7. Curcumin/Nanocurcumin Effect on Alkaline Phosphatase in Aluminum Phosphide Toxicity

Serum AP levels were significantly decreased in the ALP+Cur group compared to the ALP group (*P* < 0.05), but no significant change was observed in the ALP+Nanocur group when compared to the control group (*P* > 0.05). There was no significant difference among the ALP+Cur, ALP+Nanocur, and control groups in terms of serum ALP (*P* > 0.05) (Figure 2(c)).

### 3.8. Curcumin/Nanocurcumin Effect on Bili.T in Aluminum Phosphide Toxicity

Serum Bili.T levels were significantly decreased in the ALP+Cur (*P* < 0.01) and ALP+Nanocur groups (*P* < 0.001) compared to the ALP group. Serum Bili.T levels in the ALP+Cur and ALP+Nanocur groups were not significantly different from each other and the control group (*P* > 0.05) (Figure 2-D).

### 3.9. Curcumin/Nanocurcumin Effect on TG in Aluminum Phosphide Toxicity

Serum TG levels were significantly diminished in the ALP+Nanocur groups compared to the ALP group (*P* < 0.01), but serum TG levels in the ALP+Cur group were not significantly different from the ALP group (*P* > 0.05). Serum TG levels in the ALP+Cur and ALP+Nanocur groups were significantly lower than in the control group (*P* < 0.01). Also, serum TG levels were significantly lower in the ALP+Nanocur group than in the ALP+Cur group (*P* < 0.05) (Figure 3(a)).

### 3.10. Curcumin/Nanocurcumin Effect on T. Chol in Aluminum Phosphide Toxicity

Serum T. Chol level in the ALP+Cur and ALP+Nanocur groups was significantly lower than that of the ALP group (*P* < 0.01). Serum levels of T. Chol in the ALP+Cur group were significantly higher than the control group (*P* < 0.05), but the ALP+Nanocur group had no significant difference from the control and ALP+Cur groups in terms of T.Chol levels (*P* > 0.05) (Figure 3(b)).

### 3.11. Curcumin/Nanocurcumin Effect on VLDL in Aluminum Phosphide Toxicity

Serum VLDL levels were significantly decreased in the ALP+Cur (*P* < 0.05) and ALP+Nanocur (*P* < 0.001) groups compared to the ALP groups. Serum VLDL level in the ALP+Cur group was significantly higher than control (*P* < 0.001) and the ALP+Nanocur (*P* < 0.01) groups, but there was no significant difference between the control and ALP+Nanocur groups (*P* > 0.05) (Figure 3(c)).

### 3.12. Curcumin/Nanocurcumin Effect on HDL in Aluminum Phosphide Toxicity

In the ALP+Cur (*P* < 0.01) and ALP+Nanocur (*P* < 0.001) groups, serum HDL levels were significantly increased when compared to the ALP group. Serum HDL levels in the ALP+Cur and ALP+Nanocur groups were not significantly different from each other and the control group (*P* > 0.05) (Figure 3(d)).

### 3.13. Curcumin/Nanocurcumin Effect on LDL in Aluminum Phosphide Toxicity

In the ALP+Cur (*P* < 0.05) and ALP+Nanocur groups (*P* < 0.01), serum LDL levels were significantly lower than that of the ALP group. Serum LDL levels in the ALP+Cur group was considerably higher than that of the control group (*P* < 0.01), but there was no significant difference between the ALP + Nanocur and control groups in term of LDL (*P* > 0.05) (Figure 3(e)).

### 3.14. Curcumin/Nanocurcumin on *SIRT1*, *FOXO1a*, *FOXO3a*, *CAT* and *GPX* genes expression in Aluminum Phosphide Toxicity

Study results showed that *SIRT1*, *FOXO1a*, *FOXO3a*, *CAT* and *GPX* genes were significantly altered in the ALP group compared to the healthy control group (*P* < 0.05). Compared to controls, nanocurcumin-treated mice showed improved expression of *SIRT1*, *FOXO1a*, *CAT*, and *GPX* genes and curcumin-treated mice showed enhanced expression of *SIRT1*, *FOXO1a* genes (*P* < 0.05) (Figure 4).

### 3.15. Curcumin/Nanocurcumin Effect on Histopathological Changes in Aluminum Phosphide Toxicity

As shown in figure 5(a), hepatocytes are arranged in a radial arrangement relative to the central vein, and sinusoids are between them. Curcumin administration alone seems to cause mild dilation of sinusoids and necrosis of some hepatocytes (Figure 5(b)). Also, administration of nanocurcumin alone leads to partial central vein congestion, infiltration, and necrosis (Figure 5(c)). Severe periportal necrosis was observed in the ALP poisoned group (Figure 5(d)). Although the administration of curcumin and ALP did not positively affect the extent of damage (Figure 5(e)), administration of nanocurcumin along with ALP reduced the number of necrotic cells and central vein congestion severity (Figure 5(f)).

## 4. Discussion

Numerous biochemical tests are available as liver function markers, such as AST, ALT, AP, total bilirubin level, etc. ALT Cytoplasmic enzymes are significant markers of liver cell damage [40]. The antioxidant and hepatoprotective properties of plant extracts are evident. Lyophilized extract of *Rhus coriaria* L. is shown to be an effective antioxidant and hepatoprotective for diabetes, diabetes-related complications, and for increasing lipid profile and MDA in diabetes patients. By inhibiting lipid oxidation or reducing the production of ethanol-induced free radicals, walnuts could be valuable as diet-derived antioxidants to prevent the oxidative damage in rats. Furthermore, it can adjust AST, ALT, and LDH to prevent oxidative damage to tissues. Thus, in the tissues, ethanol-induced imbalances between MDA and fluctuating antioxidants were restored toward close control groups. Sweet gum oil was shown to have a hepatoprotective effect and antioxidant abilities against carbon tetrachloride toxicity in another study as evidence for antioxidant and hepatoprotective properties of plant extracts. Moreover, Syrian mesquite plant (*Prosopis farcta*), *Urtica dioica* Seed Extract, southern grape hyacinth, and Horse mushroom were shown to protect the liver against toxins and diseases as well as to possess antioxidant and protective properties. As seen in our earlier research, compared to controls, ALP caused a considerable rise in TAC levels, a major fall in TTG levels, a significant drop in SOD levels, a big drop in catalase activity, and a significant deterioration in mitochondrial viability. Besides, nanocurcumin treatment increased mitochondrial viability, SOD, TAC, and TTG levels. Furthermore, our current study showed a significant increase in serum AST and ALT levels in the ALP group compared to the control group [40]. The rate of change in ALT levels was much greater than that of AST, and this may be in terms of the higher sensitivity and specificity of ALT than AST for liver injury [41, 42]. Aragon et al. showed that hepatic enzymes such as ALT, AST, and ALP are released into the bloodstream due to hepatocyte cell membrane damage [43] and liver toxicity conditions [44]. As a result of ALP toxicity in rats, Yousef et al. [45] found that serum levels of AST and ALT enzymes increased. Thus, Akkaoui et al. [46], Frangides et al. [47] found that liver transaminases were elevated when ALP induced hepatotoxicity.

ALP poisoned rats had significantly increased levels of MDA, an oxidative biomarker of lipid peroxidation. Moreover, after ALP-induced toxicity, TAC dramatically reduced. As a result, oxidative stress and changes in the antioxidant defense system resulted in tissue damage caused by ALP. In contrast to the controls, the LPO levels and TAC levels in the ALP group were significantly higher in our prior work at the mitochondrial level [12]. Our present findings showed that the administration of curcumin/nanocurcumin and ALP could significantly reduce AST, ALT, and MDA and significantly increase TAC. The ability of nanocurcumin to inhibit elevated levels of ALT and MDA was greater than that of free curcumin. However, in the case of AST and TAC, curcumin and nanocurcumin had similar effects. Based on previous studies, the protective mechanism of curcumin/nanocurcumin appears to be in terms of antioxidant, anti-inflammatory and antiapoptotic properties. Corson et al. showed that curcumin inhibits hepatotoxin-induced elevated serum transaminases by inhibiting the secretion of inflammatory factors TNF-*α* and interleukin-1 from macrophages [48]. Curcumin exerts its anti-inflammatory effect via the JAK-STAT signaling pathway [49]. In Farzanegi et al. study, decreased activity of AST and ALT enzymes in the damaged liver after curcumin consumption was due to its antioxidant properties [50]. It has been found that beta-diketone phenolic groups and methoxy groups in curcumin are responsible for its antioxidant properties [51]. Curcumin's inhibitory impact on increased AST and ALT enzymes in hepatotoxic circumstances was shown to be due to its antiapoptotic action (Bax reduction and Bcl2 induction) by Shahsavan et al. [52]. Some studies have also shown that curcumin improves liver function and, as a result, leads to lower hepatic enzymes in the blood [53]. The more significant effect of nanocurcumin on ALT inhibition than curcumin in the present study could be in terms of lower solubility and lower curcumin bioavailability than nanocurcumin. Nanocurcumin can overcome many limitations of curcumin [54]. In contrast to our results, Clarke et al. showed that curcumin supplementation did not significantly affect the levels of biochemical markers in liver fibrosis models [55]. The serum ALP and total bilirubin levels were significantly increased in the ALP poisoned group. Curcumin inhibited the increase in total bilirubin and mainly elevated in serum in terms of bile duct congestion and functional impairment of damaged liver cells. Increased bilirubin levels also indicate ALP poisoning mentioned in studies [56, 57]. A decrease in serum ALP and total bilirubin levels in models of ALP-induced hepatotoxicity was reported in Sreepriya and Bali's [58] and Pari and Amali's. [59] studies. Curcumin/nanocurcumin can inhibit the release of intracellular hepatic enzymes into the blood by restoring cell membrane integrity and hepatocyte regeneration. According to the results of the current research, rats with hepatotoxicity brought on by ALP had higher levels of triglycerides, cholesterol, LDL, and VLDL, but their HDL levels were lower. ALP and curcumin coadministration had no impact on triglyceride levels. When compared to the control group, the cholesterol, LDL, and VLDL levels in the curcumin group were still much lower than those in the ALP-poisoned rats, despite curcumin's dramatic reduction in cholesterol, LDL, and VLDL and rise in HDL. However, the administration of nanocurcumin led to the return of cholesterol, LDL, VLDL and HDL to normal levels. In the case of triglyceride, nanocurcumin only caused a significant decrease, but the reduction was insufficient to restore normal levels [60]. According to previous studies, disruption of lipid metabolism in animal hepatotoxicity models may be in terms of hepatocellular injury, decreased lipase activity, impaired uptake of LDL-C and HDL-C by monocytes and macrophages, and etc. [60]. The positive effect of curcumin/nanocurcumin on regulating plasma lipid profile in rats with hepatotoxicity is consistent with the Kamalakkannan et al. study. They indicated that the lipid-lowering effect of curcumin on liver toxicity is mainly in terms of the antioxidant properties of curcumin and its preventing effect on membrane fatty acid degradation/release. Another possible mechanism was improving the impact of curcumin on liver function [61]. Nakagawa et al. showed that curcumin enhances lipid uptake by cells [62]. According to Zhou et al.'s study, curcumin increases HDL by cholesteryl ester transfer protein (CETP) inhibition [63]. It also inhibits the absorption of lipids from the digestive system and HMGCOA reductase and fatty acid synthase enzymes [64, 65]. The genes expressed in this study show that ALP can disrupt oxidative modulators at the level of gene expression, which is in line with the study of Afolabi et al. [66]. An exposure to ALP lowers the level of GSH and the total antioxidant capacity and CAT and GPX [67, 68]. Moreover, it is reported to SOD and MDA levels [69]. The histopathologic findings confirmed the biochemical results. In the ALP-poisoned group, severe periportal necrosis was observed. These observations were consistent with Anand et al. [68] and Yousef et al. [45] findings. Although mild damage was observed in the histopathological results of the curcumin/nanocurcumin alone treated groups, the damage severity was insufficient to alter the serum parameters level. Our research is in line with that of Heydari et al., who observed liver damage in pathological results but did not identify any significant changes in the levels of the enzymes AST, ALT, and ALP [70]. According to histopathological findings, there was no good protective impact on liver toxicity-induced damage in the ALP+Cur group. This can be at odds with what the serum results show. However, studies showed that necrosis does not necessarily coincide with the release of aminotransferases and the absolute increase in aminotransferases in acute liver disorders does not have prognostic significance [70]. Histopathologic findings in ALP+Nanocur group reduced the number of necrotic cells at the venous congestion amount, consistent with the serum findings. This finding is consistent with the Sankar et al. [71, 72] studies.

## 5. Conclusion

This study showed that ALP-induced hepatotoxicity in male rats significantly increased the levels of ALT, AST, and ALP enzymes, and total bilirubin, cholesterol, triglyceride, LDL VLDL, and MDA. On the other hand, ALP-induced hepatotoxicity resulted in a significant decrease in HDL and TAC. Most biochemical parameters were returned to normal levels after curcumin/nanocurcumin administration, such as in the control group. Curcumin was less efficient than nanocurcumin at controlling the majority of biochemical parameters. Histopathological findings also confirmed the biochemical results and indicated a more significant protective effect of nanocurcumin relative to curcumin against ALP-induced hepatotoxicity.

## Figures and Tables

**Figure 1:** Comparison of serum stress oxidative biomarkers in aluminum phosphide-induced liver toxicity in male rats. Data are expressed as mean ± SD. ^∗∗^*P* ≤ 0.01 vs. Control group. ^##^*P* ≤ 0.01 vs. ALP group. ^††^*P* ≤ 0.01 difference between ALP+Cur and ALP+Nanocur groups.

**Figure 2:** Comparison of serum liver biomarkers in aluminum phosphide-induced liver toxicity in male rats. Data are expressed as mean ± SD. ^∗∗^*P* ≤ 0.01 and ^∗∗∗^*P* ≤ 0.001 vs. Control group, ^#^*P* ≤ 0.05, *^##^P* ≤ 0.01, and ^###^*P* ≤ 0.001 vs. ALP group. ^†^*P* ≤ 0.05 and ^††^*P* ≤ 0.01 difference between ALP+Cur and ALP+Nanocur groups.

**Figure 3:** Comparison of lipid profiles in aluminum phosphide-induced liver toxicity in male rats. Data are expressed as mean ± SD. ^∗^*P* ≤ 0.05, ^∗∗^*P* ≤ 0.01, and ^∗∗∗^*P* ≤ 0.001 vs. Control group, ^#^*P* ≤ 0.05, *^##^P* ≤ 0.01, and ^###^*P* ≤ 0.001 vs. ALP group. ^†^*P* ≤ 0.05 and ^††^*P* ≤ 0.01 difference between ALP+Cur and ALP+Nanocur groups.

**Figure 4:** The expression of SIRT1, FOXO1a, FOXO3a, CAT, and GPX genes in the study groups. Data are reported according to mean ± SD: C: control; ALP: aluminum phosphide; Cur: curcumin; Ncur: nanocurcumin. A: significant compared to healthy control group; b: significant compared to the poisoned control group (^∗^*P* < 0.05, ^∗∗^*P* < 0.01).

**Figure 5:** Histopathological evaluation of liver tissue in ALP-poisoned male rats using hematoxylin-eosin staining. (a) Control group, (b) curcumin group, (c) nanocurcumin group, (d) aluminum phosphide group, (e) ALP+Cur group, (f) ALP+Nanocur group. H: hepatocytes; CV: central vein; Syn: sinusoids; Inf: infiltration; and Nec: necrosis.

## Data Availability

Data is available with the corresponding request.
